# Subjective evaluation of monopolar radiofrequency treatment by patients in aesthetic rejuvenation

**DOI:** 10.1111/srt.13593

**Published:** 2024-01-26

**Authors:** Yousun Hwang, Smith Arayaskul, Vasanop Vachiramon, Kyu‐Ho Yi

**Affiliations:** ^1^ Haedrin Clinic Center for Aesthetic Medicine Seoul Republic of Korea; ^2^ Smith Prive' Aesthetique Bangkok Thailand; ^3^ Department of Internal Medicine Faculty of Medicine Ramathibodi Hospital Mahidol University Bangkok Thailand; ^4^ Maylin Clinic (Apgujeong) Seoul Republic of Korea; ^5^ Division in Anatomy and Developmental Biology Department of Oral Biology Human Identification Research Institute BK21 PLUS Project Yonsei University College of Dentistry Seoul Republic of Korea

**Keywords:** anti‐aging, facial rejuvenation, monopolar RF treatment, patient evaluation, radiofrequency treatment, subjective assessment

## Abstract

**Objective:**

To assess the subjective experiences of patients following monopolar radiofrequency (RF) treatment for facial rejuvenation and anti‐aging purposes.

**Methods:**

A study involving 50 female patients (aged 30–70 years, Fitzpatrick skin type III and IV) who received a single session of RF treatment. Exclusion criteria comprised active infections, skin diseases, pregnancy, or history of recent anti‐aging treatments. Thirty‐four patients completed a 10‐question questionnaire after 3 months of treatment.

**Results:**

Among the respondents, 82% expressed satisfaction with the RF treatment, reporting significant improvements primarily in the mid and lower face, and eyelids. Mainly, patients noted improvements in skin laxity (52.9%), skin texture (17.6%), and skin tone (11.7%). Notably, 73.5% noticed changes within 1–2 months post‐treatment, with the peak effect observed at 1–2 months. Mild complications (swelling and erythema) were reported, usually resolving within a week. The mean pain score was 1.94 (±0.66), indicating mild to moderate discomfort.

**Discussion:**

Monopolar RF devices, apply high‐frequency electric currents generating heat, stimulating collagen production for skin tightening. This study's unique focus on detailed subjective patient experiences provides insights valuable in clinical settings, aiding clinicians in managing patient expectations and achieving optimal results. The satisfaction rates align with previous findings, emphasizing RF treatment's efficacy in addressing facial laxity, especially in the mid and lower face. Positive feedback extended beyond skin tightening, encompassing skin texture and tone improvements. While the study's observation period was 3 months post‐treatment, longer‐term studies are warranted for comprehensive assessments.

**Conclusion:**

The study underscores the efficacy of monopolar RF device, as a non‐invasive and effective anti‐aging treatment. The findings contribute to diversifying the RF market, potentially aiding clinicians in optimizing patient care. Considering the growing complexity of patient demands and treatment responses, this study serves as a valuable reference for clinicians engaging in RF treatments.

## 1 INTRODUCTION

For a considerable duration, cosmetic surgery has remained the cornerstone of Aesthetic Medicine. Nonetheless, concerns regarding significant side effects and prolonged recovery periods have spurred a shift towards less invasive methods. This surge in demand for innovative approaches has led to notable advancements in technologies. Conventional techniques like ablative lasers and chemical peels have evolved into more sophisticated methods such as fractional laser, radiofrequency (RF), and high‐intensity focused ultrasound (HIFU) treatments, all aiming to offer more natural results while minimizing downtime.^1^

Monopolar RF devices possess a unique feature: the high‐frequency electric current they generate produces heat capable of penetrating the deep dermal layers and fat tissues while safeguarding the epidermis. This heating process has been associated with the alteration of collagen, resulting in its thickening and shortening, thereby gradually tightening the skin over a span of 4–6 months.^2^

Numerous studies have sought to explore the effects of RF treatment, employing histologic analysis,^2^ patient assessments,^3^ and evaluations conducted by impartial physicians.^4^ While these studies have generally reported favorable outcomes, their assessments have often centered on specific criteria, such as the Global Aesthetic Improvement Scoring system, Fitzpatrick Wrinkle Classification, and Laxity Classification.^4^

Our study aims to delve deeper by gathering more comprehensive feedback from patients following RF treatment. This endeavor is crucial in clinical settings, offering valuable insights for clinicians to better anticipate and understand patients' experiences. To achieve this goal, we conducted a survey involving 34 patients and administered a 10‐question questionnaire tailored to assess their RF treatment outcomes.^1^

## 2 METHOD

Fifty female participants aged between 30 and 70 years, exhibiting mild to moderate facial sagging and categorized as Fitzpatrick skin types III and IV, received a single session of RF (Radiofrequency) treatment using the Volnewmer device from Classyc Inc. Korea, between March 1, 2023, and August 31, 2023. Exclusion criteria encompassed active infections, skin diseases, history of keloidal scarring, pregnancy, or undergoing any anti‐aging treatment within the past 6 months. All participants provided informed consent upon enrollment and agreed to complete a questionnaire 3 months post‐treatment, although only 34 participants returned the completed questionnaire.

Following informed consent, participants' faces were cleansed, and without the application of topical anesthetic cream, 300 shots were administered to the entire face using an initial energy level of 3 J/cm^2^, which was reduced to 2.5 in cases where participants reported severe pain during the procedure. Post‐treatment, participants returned home. The questionnaire, comprising 10 questions, was sent to each participant 3 months after the treatment, primarily consisting of multiple‐choice questions, with an option for participants to provide subjective answers when applicable.

One of the questions asked participants to rate their overall satisfaction on a 0–4 scale using the Global Aesthetic Improvement Scoring system, which defines the levels of improvement from “Very much improved” to “Worsened.” Participants also rated their pain levels based on the Verbal Rating Scale (VRS) from 0 to 3, ranging from “No pain or discomfort” to “Severe pain,” characterized by verbal responses, facial expressions, or tears.

The questionnaire included inquiries regarding the level of improvement, specific areas of satisfaction on the face, aspects of change satisfaction, the timeline for noticing changes and peak effects, pain during treatment, any adverse effects post‐treatment, downtime duration, willingness to undergo treatment again, and concerns if opting for the treatment in the future (Figure 1).

**FIGURE 1:** Participants were asked to rate the improvement level on a scale from 1 to 5, specify the facial area they were most satisfied with if their score was below 4, identify the aspect of change they were most content with, report when they first noticed the treatment's effects, indicate when they felt the maximum effect, describe the intensity of pain during treatment using a scale of 0–3, disclose any post‐treatment unwanted effects, state the duration of downtime, express their willingness for retreatment, and pinpoint their primary concern if considering the treatment again.

## 3 RESULTS

Out of the 50 patients who underwent the treatment, 34 successfully completed the study, with ages ranging from 36 to 66 years (mean: 49.21 ± 7.91 years). Among them, 23 patients exhibited Fitzpatrick skin type III, while 11 had Fitzpatrick skin type IV. Impressively, over 80% (82%) of the individuals treated with RF expressed satisfaction with the outcomes. The average Global Aesthetic Improvement Scale (GAIS) score stood at 2.71 ± 0.87 (Figure 2). Notably, participants reported the most significant improvements in the mid‐face (13 patients; 38.2%), lower face (12 patients; 35.2%), and eyelids (three patients; 8.8%), with no notable improvements reported on the forehead. Skin laxity enhancement was identified as the most noticeable change (18 patients; 52.9%), followed by improvements in skin texture (six patients; 17.6%) and skin tone (four patients; 11.7%). Around 73.5% of patients (25 patients) noticed differences after 1–2 months (15 patients; 44%) or at 3 months (three patients; 8.8%), while 29.4% (10 patients) observed changes immediately after treatment. The peak effect was observed at 1–2 months by 52.9% (18 patients) and at 3 months by 20.6% (seven patients), with 8.8% (three patients) experiencing the greatest effect in less than a month. A majority (55.9%) reported no treatment‐related complications, although mild issues like swelling (nine patients; 26.5%) and erythema (six patients; 17.6%) occurred, usually resolving within a week (12 patients; 35.3%) or a month at most (three patients; 8.8%). The mean pain score was 1.94 (± 0.66), indicating mild to moderate pain during the procedure. Nonetheless, 61.7% (18 patients) expressed their willingness to undergo the treatment again, with the primary concern for the next treatment being pain (14 patients; 41.2%), followed by concerns about the treatment's effectiveness (10 patients; 29.4%).

**FIGURE 2:** The figure illustrates the Global Aesthetic Improvement Scale (GAIS) scores, ranging from 1 to 5, denoting: (1) Very much improved, (2) Much improved, (3) Somewhat improved, (4) Unchanged, and (5) Worsened.

Radiofrequency (RF) technology employed in skin rejuvenation operates within an electromagnetic frequency spectrum spanning from 0.5 to 40 MHz. Tissue impedance to electrical currents generates heat, and the energy can be computed using the formula: Energy (J) = I^2 × R × T (where I represents Current, R denotes Impedance, and T signifies Time in seconds).^5^ The correlation between heat production, electrical current potency, and tissue resistance yields varying outcomes across different tissues and individuals. Following the market introduction of Thermacool (Solta Medical, Inc., formerly Thermage, Hayward, CA, USA) for skin tightening and facial wrinkle treatment, numerous RF devices emerged, each embracing slightly varied technologies. Among these, Volnewmer, a monopolar RF device manufactured by Classys Inc. in South Korea, shares comparable frequency (6.78 MHz) and power (watt) with Thermacool but distinguishes itself through several noteworthy features. Its convex‐shaped tip, adaptable to surface angles, facilitates uniform energy dispersion into the dermis while ensuring steadfast surface attachment. Moreover, its innovative cooling mechanism employing water instead of gas provides instant surface cooling, reducing pain during treatment while effectively delivering RF energy into the deeper dermis.

The choice between monopolar and bipolar radiofrequency therapies hinges on treatment objectives, targeted skin regions, and the desired skin penetration depth. Palmieri et al.^6^ indicated that monopolar electrodes exhibit deeper penetration into skin layers, reaching subcutaneous tissues for substantial collagen remodeling, which is crucial in skin rejuvenation treatments aiming for comprehensive tightening effects. They're also versatile, applicable to various body areas. Monopolar RF excels in treating larger areas and achieving profound skin tightening by penetrating deeply into subcutaneous tissues, enabling substantial collagen remodeling. Its versatility allows application across various body areas and offers notable clinical improvements, especially in addressing mild to moderate wrinkles or post‐lifting concerns. Conversely, bipolar RF, while precise and safer for delicate areas, may have limitations in penetration depth and coverage area, potentially resulting in less pronounced effects, particularly for extensive skin tightening or larger treatment zones.^6^, ^7^, ^8^

Diverse evaluation methodologies have been employed to gauge RF treatment efficacy. Subjective assessments,^9^, ^10^ histopathological evaluations,^11^, ^12^ and radiological appraisals^13^ have all been utilized to appraise outcomes. Most subjective findings underscore the clinical significance of RF treatment,^9^, ^10^ while histopathological analyses demonstrate heightened collagen synthesis.^11^, ^12^ This study, unlike prior research, prioritized a comprehensive exploration of patients' subjective experiences through a detailed questionnaire. This approach, within clinical settings, aids clinicians in understanding patients' nuanced needs, establishing realistic expectations, and attaining more optimal results.

The satisfaction rate among subjects was notably high, albeit the reasons behind their ratings varied. Notably, the mid‐face and lower face garnered the most satisfaction, aligning with prior research underscoring RF treatment efficacy for middle and lower face laxity.^14^, ^15^, ^16^ Plausibly, this could relate to the treatment's impact on subcutaneous fat tissue, contributing to volume loss around marionette lines and an overall slimming effect. Furthermore, the Energy(J) = I^2^ × R × T equation posits that, given the higher impedance of fat compared to the skin or muscle, the lower face, being relatively more fat‐dominant than the forehead, might receive higher penetrating energy, potentially explaining the observed outcomes. Although RF treatment can benefit eyelid sagging, none reported improvements in forehead appearance.^17^

Additionally, it is crucial to note that positive feedback extended beyond skin tightening to include skin texture and tone. RF treatment typically yields gradual improvements; while this study observed peak improvement at 1–2 months post‐treatment, previous research has reported significant enhancement at 3 and 6 months post‐treatment.^18^ Nonetheless, longer follow‐up periods beyond 3 months would offer deeper insights.

Most patients exhibited tolerance to mild to moderate pain, as reflected in the Verbal Rating Scale (VRS) used in this study instead of the Numerical Rating Scale (NRS) for its simplicity and high correlation with NRS, ensuring higher response rates.^19^ Reported complications, such as swelling and erythema, dissipated within a month, affirming the non‐invasive nature of the treatment. Interestingly, the study revealed that treatment cost did not emerge as a primary concern, which contrasts with prior research highlighting price as a significant consideration among female Asian patients.^20^, ^21^

The enduring quest for enhanced physical appearance, epitomized by the popularity of plastic surgeries in the 21st century, has evolved with the advent of less invasive techniques. However, meeting patients' intricate needs in this multifaceted landscape remains challenging. Though critiques persist regarding the subjective basis of some influential RF treatment studies,^22^ subjective assessments remain crucial, representing the voices of patients that clinicians encounter daily. As the RF device market expands annually, understanding patients' nuanced responses and concerns equips clinicians with the confidence to provide more tailored treatments.

Limitations of the study conducted on Radiofrequency (RF) treatment in skin rejuvenation include the relatively small sample size, with only 34 out of 50 participants completing the survey, potentially limiting the representativeness of the findings. The study focused on female participants aged between 30 and 70 years with mild to moderate facial sagging, which may restrict the generalizability of the results to other age groups or individuals with different skin concerns. Additionally, the research utilized a single device, the Volnewmer from Classyc Inc., which may not account for variations in outcomes that could arise from using different RF devices or technologies. Moreover, while the questionnaire method offered subjective feedback from participants, it may introduce response biases or limitations inherent to self‐reported data. Lastly, the absence of a control group or comparative analysis with alternative treatments could restrict a thorough assessment of RF treatment efficacy in relation to other available modalities.

Cosmetic procedures, while offering aesthetic enhancements, pose challenges in catering to diverse patient needs. Our study exploring patients' subjective responses to RF treatment via a questionnaire underscores monopolar RF effectiveness as a non‐invasive anti‐aging treatment. This finding broadens the horizon of the burgeoning RF market and stands as a reference for clinicians actively engaged in RF treatments.

## CONFLICT OF INTEREST STATEMENT

There is no conflict of interest for all authors.

## Data Availability

The author has provided the required Data Availability Statement, and if applicable, included functional and accurate links to said data therein.
